RETRACTED

# Comparison of Dexmedetomidine and Etomidate on Intraoperative Wake-Up Equality, Hemodynamics, and Cerebral Protection in Operation of the Brain Functional Area

**DOI:** 10.1155/2021/6363188

**Published:** 2021-08-26

**Authors:** Yuerong Peng, Qinglai Guan

**Affiliations:** Department of Anesthesiology, Huashan Hospital, Fudan University, No. 12, Middle Wulumuqi Road, Shanghai 200040, China

## Abstract

In recent years, with the increasing incidence of brain functional area tumors, the clinical application of functional area tumor resection has become extremely urgent. Intraoperative wake-up is an important auxiliary method of this operation, which can effectively reduce the damage of the brain function area caused by the operation and anesthesia itself while playing the role of auxiliary function area and tumor positioning. However, the intraoperative wake-up requires a higher anesthesia effect, so higher requirements are put forward for the choice of anesthetic drugs. Based on hemodynamic and serum molecular observations, this study found that dexmedetomidine- and etomidate-assisted anesthesia were used for intraoperative wake-up in brain functional area surgery, both of which could maintain hemodynamic stability. In addition, the arousal effect and brain protection of dexmedetomidine were better than those of etomidate, and the incidence of adverse reactions was lower during the arousal period. This can provide relevant reference for clinical improvement of the anesthesia effect and surgical safety of intraoperative wake-up.

## 1. Introduction

The operation risk of brain functional lesions is extremely high because the normal brain tissue is easy to be damaged in conventional operation. It can result in neurological impairment, which may involve the patients with language, sensory, or limb disorders after the operation [1]. The intraoperative wake-up technique is one of the important auxiliary techniques for brain functional area tumor resection. It can keep the patient under a certain analgesic and sedative state and clear consciousness to cooperate with the doctor to complete the functional area positioning, which optimizes the operation result of surgical resection and reduces the damage that may happen to the normal brain functional area [2]. To ensure the smooth development of this procedure, during the awakening period of the surgery, in addition to ensuring that the patient has a clear cognition, avoiding severe hemodynamic changes, and maintaining a stable breathing state, it is also necessary to ensure that the patient has a good anesthesia and analgesic effect, so that it can cooperate with the surgery to the greatest extent. Physician's positioning of the functional areas of the brain improves compliance with surgical treatment [3, 4]. However, in clinical practice, since anesthesia itself can have varying degrees of impact on the patient's neurological function and hemodynamics, the intraoperative wake-up technique for brain functional area surgery puts forward higher requirements for effectiveness and safety for the application of anesthetics. Etomidate is a nonbarbiturate narcotic drug with fast onset and high safety factor and has little effect on the respiratory and circulatory systems [5]. Dexmedetomidine does not act on the cerebral cortex, nor cause respiratory depression with the characteristics of “awake sedation,” which showed it is suitable for arousal anesthesia [6, 7]. In this study, dexmedetomidine and etomidate were, respectively, used for intraoperative wake-up in brain functional areas, aiming to compare the intraoperative wake-up effects of the two and to observe the effects on hemodynamics and brain protection. The details are as follows.

RETRACTED

## 2. Materials and Methods

### 2.1. General Information

A total of 74 patients, 41 males and 33 females, aged from 18 to 60 years, with an average age of 48.54 ± 16.38 years, who underwent brain functional area surgery in our hospital from February 2018 to June 2019 were selected. Inclusion criteria: age ≥18 years; the lesions confirmed by CT and MRI examination required intraoperative wake-up-assisted surgical resection; American Association of Anesthesiologists (ASA) I∼II rated; and met the indications of surgery, anesthesia, and intraoperative wake-up. Exclusion criteria: contraindication of surgery or related drugs; severe cardiopulmonary insufficiency; history of hypertension; complicated with serious diseases of the immune system and blood system; pregnant or lactating women; and cognitive dysfunction. Etiology: glioma in 43 cases; meningioma in 31 cases. According to the random number table method, the patients were divided into the observation group (*n* = 37) and the control group (*n* = 37). There was no statistical difference in general data between the two groups (*P* > 0.05), as shown in Table 1. This study was approved by the ethics committee of our hospital, and all patients or their families gave informed consent and signed the informed consent.

### 2.2. Treatment Methods

Both groups were treated with general anesthesia-assisted intraoperative wake-up for surgical excision. Induction of general anesthesia: An appropriate amount of remifentanil (Yichang Renfu Pharmaceutical Co., Ltd., National Medicine Standard H20054171), propofol (Zhejiang Jiuxu Pharmaceutical Co., Ltd., National Medicine Standard H20084531), and cis-atracurium (Jiangsu Hengrui Pharmaceutical Co., Ltd., National Medicine Standard H20060869) was given intravenously, the endotracheal catheter was placed to assist mechanical ventilation, and tidal volume 8–10 ml/kg, respiratory rate 10–20 times/min, and 35–40 mmHg of CO_2_ partial pressure at the end of expiration were maintained. Anesthesia maintenance: remifentanil 2.0 ng/mL and propofol 2.5 *μ*g/mL were adjusted; meanwhile, the observation group was given dexmedetomidine (Jiangsu Hengrui Pharmaceutical Co, Ltd., National Medicine Standard H20090248) 1.0 *μ*g/mL loading dose, which was adjusted to 0.5 *μ*g/kg/h infusion 10 min later. The control group was given etomidate (Jiangsu NHWA Pharmaceutical Co., Ltd, National Medicine Standard H32022992) infusion of 10.0 *μ*g/kg/h. During the surgery, blood pressure was maintained at the base value of ±30% and heart rate was maintained 50–100 beats/min, and dopamine or atropine was given when necessary. Intraoperative wake-up: 10 minutes before wake-up, remifentanil was adjusted to 0.5 ng/ml, dexmedetomidine was adjusted to 0.2 *μ*g/kg/h in the observation group, and etomidate infusion was stopped in the control group. After the patient resumed spontaneous breathing, his or her name was called every 30 seconds with the expectation to receive response and the patient was asked to move his or her hands and feet. When the patient was able to respond without mistake, it was deemed that the arousal was successful. While the patient remained awake, intraoperative neuronavigation and cortical microelectric stimulation were combined to complete the localization of the lesion, followed by reanesthesia and surgical resection under a microscope.

RETRACTED

### 2.3. Observation Indicators

The wake-up time, recovery time of spontaneous respiration, and recovery time of directional force of patients were recorded. The mean arterial pressure (MAP), heart rate (HR), and blood oxygen saturation (SPO_2_) of the patient were recorded at 30 min before arousal (T1), the beginning of arousal (T2), successful arousal (T3), 15 min after successful arousal (T4), and 10 min after reanesthesia after arousal (T5). The adverse reactions of the two groups during intraoperative arousal were recorded, including tachycardia (heart rate >100 beats/min), bradycardia (<50 beats/min), hypertension (≥130% of the baseline value), hypotension (≤70% of the baseline value), coughing with physical activity, respiratory depression, nausea and headache, and wake-up memory after surgery. Before and 24 h after surgery, 5 ml of venous blood was extracted from both groups. Serum levels of S100*β* protein and neuron-specific enolase (NSE) were detected by enzyme-linked immunoassay. The kits were purchased from Shanghai Enzyme-linked Biotechnology Co., Ltd.

RETRACTED

### 2.4. Statistical Methods

The SPSS22.0 was adopted to process data. The measurement data were expressed as mean ± standard deviation ($\bar{x}$ ± s), the analysis of variance was used for comparison, and the SNK method was used for pairwise comparison. The count data were expressed as rate (%), and *χ*^2^ test was implemented; *P* < 0.05 indicated that the difference was statistically significant.

## 3. Results

### 3.1. Comparison of the Effects of Intraoperative Arousal between the Two Groups

The intraoperative wake-up time, recovery time of spontaneous respiration, and recovery time of directional force in the observation group were all shorter than those in the control group (*t* = 4.838, *P* < 0.001; *t* = 6.295, *P* < 0.001; and *t* = 2.869, *P*=0.005), as shown in Figure 1.

### 3.2. Comparison of Hemodynamic Indexes between the Two Groups

There was no statistical difference between the two groups of MAP and SPO2 at the time points of T1, T2, T3, T4, and T5 (*P* > 0.05). At each time point of T1, T2, T3, T4, and T5, the HR of the observation group was lower than that of the control group at the same time point (*P* < 0.05). At T2, HR in both groups was higher than T1 in the same group; at T3, the HR of the control group was higher than T1 and T2 of the same group, and the HR of the observation group was higher than T1 of the same group; at T4, the HR of the control group was higher than T1 and T2 of the same group, and the HR of the observation group was higher than T1, T2, and T3 of the same group; at T5, HR in the control group was lower than that at T2, T3, and T4, while HR in the observation group was higher than that at T1 and lower than that at T2, T3, and T4 (*P* < 0.05), as shown in Table 2.

### 3.3. Comparison of Brain Injury Indexes between the Two Groups

Serum levels of S100*β* protein and NSE 24 h after surgery in the observation group were lower than those in the control group and 24 h after surgery in both groups were higher than those before surgery (*t* = 3.965, *P* < 0.001; *t* = 2.997, *P*=0.004), as shown in Figure 2.

### 3.4. Comparison of Adverse Reactions during the Wake-Up Period between the Two Groups

During the wake-up period, in the control group, there were 3 cases of nausea and headache, 2 cases of tachycardia, 2 cases of cough, 1 case of hypotension, 1 case of bradycardia, 1 case of wake-up memory after surgery occurred, 10 cases in total (10/37), and the incidence of adverse reactions was 27.03%. In the observation group, there were 1 case of bradycardia, 2 cases of hypotension, 3 cases in total (3/37), and the incidence of adverse reactions was 8.11%. The incidence of adverse reactions in the observation group was lower than that in the control group (*χ*^2^ = 4.573, *P*=0.032), as shown in Figure 3.

RETRACTED

## 4. Discussion

The general anesthesia technique induces the loss of consciousness of the patient by acting on the neural circuit responsible for the sleep-wake transition, to achieve the purpose of painless surgery. But, for patients undergoing tumor resection of the brain function area, the maximum resection of the lesion should be performed under the premise of ensuring the normal functioning of important brain functions; for this, conventional anesthesia and surgical techniques cannot fully meet its requirements, since the functional areas of the brain have important physiological functions in terms of sensation, language, and movement [8]. The neuroelectrophysiological monitoring technology can monitor the changes in the electrical signals transmitted by the nerves of the brain functional areas in real time and accurately locate the cortical functional areas, thereby improving the success rate and safety of surgery and reducing neurological damage [9, 10]. Among them, the cortical microcurrent stimulation technology has high positioning accuracy, which can detect both cortical function and subcortical conduction pathways [11]. However, this technique requires the patient to remain fully awake, so it is necessary to wake up intraoperatively after general anesthesia.

The results showed the intraoperative wake-up time, recovery time of spontaneous respiration, and recovery time of directional force in the observation group were all shorter than those in the control group. This indicates that dexmedetomidine has a better effect on intraoperative wake-up than etomidate has. Analyzing the reasons, etomidate is an anesthetic widely used in clinics. It has a high binding rate to plasma proteins, can quickly pass through the blood-brain barrier to exert sedative and hypnotic effects, and has the characteristics of short half-life and fast metabolism in the body [12, 13]. Dexmedetomidine can act on the central and peripheral nerves at the same time, inhibit pain signal transduction, and produce sedation and analgesia, its half-life is also short, and the protein binding rate is higher [14, 15]. Therefore, dexmedetomidine has a better arousal effect than etomidate. Both dexmedetomidine and etomidate have low effects on the circulatory system, and both of them can maintain hemodynamic stability [16, 17]. From the result, we can conclude that there was no statistical difference in the changes of hemodynamic indicators between the two groups during the arousal period. It indicates that both the groups had a slight impact on the cardiovascular system. At each time point during the arousal period, the HR of the observation group was lower than that of the control group. The difference may be caused by the inhibition of sympathetic nerve excitement by dexmedetomidine [18]. However, from the point of view of adverse reactions, this inhibitory effect was not serious, and the incidence of adverse reactions of dexmedetomidine during intraoperative wake-up was significantly lower than that of the control group. Analyzing the reasons, this may be because dexmedetomidine has a good neuroprotective effect compared to etomidate, so it can effectively avoid the further influence of anesthesia and surgery itself on the patient.

RETRACTED

The serum levels of S100*β* protein and NSE are serological indicators closely related to central nervous system damage; among them, the former exists in glial cells, and the latter exists in neuronal cells. After the central nervous system is damaged, both are released into the blood in large quantities [19, 20]. In this study, the serum levels of S100*β* protein and NSE of the two groups at 24 h after surgery were higher than those of the same group before surgery, but the serum levels of S100*β* protein and NSE of the observation group were significantly lower than those of the control group. The abovementioned results indicate that there is a certain degree of damage to the brain tissue after surgery, and the use of dexmedetomidine for intraoperative wake-up can reduce nerve damage, improve the safety of anesthesia, and reduce the impact of surgical stimulation on the physiological functions of brain tissue such as cerebral blood flow and brain metabolism rate by inhibiting astrocyte activation and antisympathetic effect, so it has obvious protection of the brain [21, 22].

In summary, dexmedetomidine- and etomidate-assisted anesthesia brain function area surgery for intraoperative wake-up can maintain hemodynamic stability, but the effect of intraoperative wake-up and brain protection of dexmedetomidine is better than that of etomidate, the incidence of adverse reactions during the arousal period is lower, and it is suitable for clinical application.

## Figures and Tables

**Figure 1:** Comparison of the effects of intraoperative arousal between the two groups ($\bar{x}$ ± s, min). Note: the intraoperative wake-up time, recovery time of spontaneous respiration, and recovery time of directional force in the control group were (10.74 ± 2.38) min, (8.40 ± 1.66) min, and (12.45 ± 2.84) min, respectively. The intraoperative wake-up time, recovery time of spontaneous respiration, and recovery time of directional force in the observation group were (8.45 ± 1.62) min, (6.31 ± 1.15) min, and (10.69 ± 2.42) min, respectively. ^*∗*^The difference between the two groups was statistically significant.

RETRACTED

**Figure 2:** Comparison of brain injury indexes between the two groups ($\bar{x}$ ± s, *μ*g/L). (a) Comparison of S100*β* protein between the two groups. (b) Comparison of S100*β* protein between the two groups. Note: the levels of S100*β* protein were (1.09 ± 0.24) *μ*g/L and (1.92 ± 0.41) *μ*g/L before and 24 h after surgery in the control group and (1.12 ± 0.29) *μ*g/L and (1.56 ± 0.37) *μ*g/L before and 24 h after surgery in the observation group, respectively. The levels of NSE were (2.65 ± 0.55) *μ*g/L and (4.26 ± 0.67) *μ*g/L before and 24 h after surgery in the control group and (2.72 ± 0.49) *μ*g/L and (3.80 ± 0.65) *μ*g/L before and 24 h after surgery in the observation group, respectively.^*∗*^Comparison with the same group before surgery, *P* < 0.05; #comparison with the control group after surgery, *P* < 0.05.

**Figure 3:** Comparison of the occurrence of adverse reactions during the wake-up period between the two groups (cases).

**Table 1:** Comparison of general information between the two groups.

Types	Control group (*n* = 37)	Observation group (*n* = 37)	*χ*^*2*^/*t*	*P*
Gender			0.492	0.483
Male	19	22		
Female	18	15		
Age (years)	48.92 ± 14.63	48.16 ± 15.05	0.220	0.826
Etiology			0.056	0.814
Glioma	21	22		
Meningioma	16	15		

**Table 2:** Comparison of hemodynamic indexes between the two groups ($\bar{x}$ ± s).

Group	Time	MAP (mmHg)	HR (times/min)	SPO_2_ (%)
Control group (*n* = 37)	T1	96.29 ± 7.42	74.87 ± 6.54	96.06 ± 3.08
	T2	97.63 ± 7.23	85.31 ± 7.27^a^	95.73 ± 2.97
	T3	98.22 ± 6.85	90.57 ± 6.35^ab^	95.27 ± 3.68
	T4	99.47 ± 6.82	92.32 ± 5.16^ab^	95.11 ± 2.94
	T5	97.54 ± 6.65	77.24 ± 4.58^bcd^	96.02 ± 3.21
*F*		0.724	1.924	0.620
*P*		0.472	0.058	0.547
Observation group (*n* = 37)	T1	95.86 ± 7.75	68.51 ± 5.76^e^	96.14 ± 2.89
	T2	96.64 ± 7.16	74.83 ± 5.02^ae^	95.69 ± 3.25
	T3	97.59 ± 7.28	76.39 ± 4.77^ae^	95.43 ± 3.44
	T4	99.07 ± 6.74	79.67 ± 4.36^abce^	95.07 ± 2.92
	T5	96.19 ± 6.21	72.31 ± 4.05^abcde^	96.21 ± 2.88
*F*		0.500	1.660	0.439
*P*		0.654	0.101	0.645

Note: compared with T1 of the same group, ^*a*^*P* < 0.05; compared with T2 of the same group, ^*b*^*P* < 0.05; compared with T3 of the same group, ^*c*^*P* < 0.05; compared with T4 of the same group,^*d*^*P* < 0.05; compared with the control group at the same time point, ^*e*^*P* < 0.05.

## Data Availability

The original data used in this study can be obtained from the corresponding authors.
